The article "MicroRNA-217 Regulates WASF3 Expression and Suppresses Tumor Growth and Metastasis in Osteosarcoma" was retracted in 2022. Reasons: duplicated images; signs of a paper mill; unreliable results or conclusions.

# MicroRNA-217 Regulates WASF3 Expression and Suppresses Tumor Growth and Metastasis in Osteosarcoma

**DOI:** 10.1371/journal.pone.0109138

**Published:** 2014-10-07

**Authors:** Lei Shen, Peng Wang, Jili Yang, Xiaotao Li

**Affiliations:** 1 Department of Anatomy, Qiqihar Medical School, Qiqihar, Heilongjiang, China; 2 Department of Orthopedics, The Fourth Hospital of Harbin Medical University, Harbin, Heilongjiang, China; 3 Department of TCM, Jilin Province Tumor Hospital, Changchun, Jilin Province, China; 4 Department of Orthopedics, The First Affiliated Hospital of Jiamusi University, Jiamusi, Heilongjiang, China; University of Vermont, United States of America

## Abstract

Osteosarcoma is the most common type of primary tumor of bone which mainly affects adolescents and young adults. Osteosarcoma causes large number of deaths because of its complex pathogenesis and resistance to conventional treatment. MicroRNAs are a class of small noncoding RNAs that function as critical gene regulators through targeting mRNAs, causing translational repression or degradation. In this study, we showed that miR-217 was down-regulated in osteosarcoma cell lines and tissues in comparison to that in normal bone cells or tissues. Meanwhile, the lower level of miR-217 was associated with metastasis in clinical osteosarcoma patients. Furthermore, we found that overexpession of miR-217 markedly suppressed cell proliferation, migration, and invasion of osteosarcoma cells. Conversely, the inhibition of miR-217 expression significantly accelerated the cell proliferation, migration, and invasion. Moreover, we identified WASF3 as a novel functional downstream target of miR-217. The ectopic expression of WASF3 can partially reverse the inhibition of cell proliferation and invasion caused by miR-217. Take together, our results demonstrate that miR-217 functions as a tumor-suppressive miRNA and inhibits the osteosarcoma tumorigenesis through targeting WASF3.

## Introduction

Osteosarcoma is the most common type of primary sarcoma of the bone and a leading cause of cancer death in adolescents due to its rapid proliferation [1], [2]. Despite the rapid development in therapeutic strategies, such as wide tumor excision, adjuvant chemotherapy and radiotherapy, the cure rate of patients of osteosarcoma is still very low [3]. Although recent advances in molecular biology have provided some clues to the molecular pathogenesis of osteosarcoma, the exact molecular mechanisms underlying the histological heterogeneity, drug resistance, and development of metastasis remain unclear [4]. Therefore, it is urgent to develop novel targets for the diagnosis, treatment, and prognosis of osteosarcoma.

MicroRNAs (miRNAs) are a class endogenous small non-coding RNAs that regulate gene expression by the inhibition of the translation and/or decreasing of the stability of target mRNAs [5]. MiRNAs are differentially expressed in various tissues and cells, suggesting their potential applications as biomarkers and therapeutic targets [6]. MiRNAs are deregulated in several diseases including cancers, where they play important roles by regulating the expression of various tumor oncogenes and suppressors [7], [8]. MiRNAs also can act as oncogenes or tumor suppressors and involve in numerous cellular processes, playing roles in tumorigenesi by regulating cell differentiation, cell proliferation and cell cycle [9]–[13]. However, the role of miRNAs in osteosarcoma tumor development and metastasis has only recently been investigated and remains largely unknown.

Previous studies have showed that miR-217 was a novel tumor biomarker of clear cell renal cell carcinoma [14]. It could target oncogenes or tumor suppressor genes in different cell type. For example, miR-217 could target KRAS, previously shown to function as a tumor suppressor by inhibiting tumor cell growth and anchorage-independent colony formation [15]. MiR-217 could also act as oncogene by targeting the tumor suppressor gene PTEN in kidney disorders [16]. In addition, miR-217 could target silent information regulator 1 (SirT1), and function as an oncogene [17]. However, no specific study has been showed to investigate the role of miR-217 in osteosarcoma.

In this report, we investigated the role of miR-217 in human osteosarcoma. First, we investigated the expression of miR-217 in human osteosarcoma cell lines and tissues, and paired adjacent non-tumor bone tissue. Second, we examined the cell growth, migration, and invasion following overexpression or downregulation of miR-217 in osteosarcoma cell lines. Finally, we determined the target gene of miR-217 using the luciferase reporter assay and western blot.

## Materials and Methods

### Ethics Statement

All of these patients or patients' parents on behalf of the children agreed to participate in the study and gave written informed consent. Both this study and consent were approved by the ethical board of the institute of The First Affiliated Hospital of Jiamusi University and complied with the Declaration of Helsinki.

### Tissue samples

Surgically resected 60 osteosarcomas specimens and their morphologically normal bone tissues (before the administration of neoadjuvant chemotherapy) were acquired from The First Affiliated Hospital of Jiamusi University between November 2007 and November 2013. Tissue samples were cut into two parts and one part was fixed with 10% formalin for histopathological diagnosis. The other was immediately snap-frozen in liquid nitrogen and then stored at −196°C in liquid nitrogen until it was needed for RNA was extracted. The use of tissue samples for all of these experiments was approved by the patients and by the Ethics Committee of the institution. These patient characteristics were described in Table S1.

### Cell lines and Cell culture

The following human osteosarcoma cell lines were used in this study: MG-63 (14 years old, male), U2OS (15 years old, female), SOSP-9607(17 years old, male), and SAOS-2 (11 years old, female), one normal bone cell lines hFOB and 293T cells. These cell lines were purchased from the American Type Culture Collection (ATCC, Rockville, MD, USA) and were propagated in Dulbecco's modified Eagle medium (Gibco; Invitrogen; Life Technologies, Germany) that was supplemented with 10% fetal bovine serum (GIBCO, NY, USA) and streptomycin (100 µg/ml), penicillin (100 U/ml).

### Cell transfection

The miR-217 mimics, inhibitor and the scramble mimics, which were non-homologous to the human genome and were synthesized by GenePharma (Shanghai, China) and were transfected into the cells to a final oligonucleotide concentration of 20 nmol/L. All of these cell transfections were performed by DharmaFECT1 Reagent (Dharmacon, TX, USA) according to the manufacturer's instructions.

### TaqMan RT-PCR for miRNA expression

Total RNA was isolated from cultured cells or tissues samples with Trizol reagent (Invitrogen, Carlsbad, CA, USA). MiRNAs were quantitated by real-time PCR using the TaqMan MicroRNA Assays (Invitrogen, USA) [18]. First-strand complementary DNA (cDNA) synthesis was carried out using 1 µg of total RNA in a 12 µl final volume containing 2 M stem-loop primer and 10 mMdNTP Mix (Invitrogen, USA). The mix was incubated at 65°C for 5 min, and then, 5xRT buffer, 0.1 M DTT, 200 U/µl MultiScribe reverse transcriptase and 40 U/µl RNase inhibitor were added (Invitrogen, USA). Then the mix was incubated at 37°C for 55 min, followed by 70°C for 15 min, and then held at −20°C. Real-time PCR was performed using a standard TaqMan PCR protocol [18]. The 20 µl PCR reactions included 1 µl of RT product, 1× Universal TaqMan Master Mix and 1× TaqMan probe/primer mix (Invitrogen, USA). All RT reactions, including the no-template controls, were run in triplicate. All mRNA quantification data were normalized to U6 expression. The relative amount of transcript was calculated using the comparative Ct method (Table S2).

### Cell proliferation assay

Cell proliferation was analyzed by using cell counting assay Kit-8 (CCK-8) (DOJINDO, Kumamoto, Japan) according to the manufacture's protocol. Cells were incubated in 10% CCK-8 diluted in normal culture media at 37°C until the visual color conversion occurred. Proliferation rates were determined at 0, 24, 48, 72 and 96 hours after transfection. The absorbance of each well was measured with a microplate reader set at 450 nM and 630 nM.

### Cell migration and invasion assays

MG-63 cells were grown to confluence in 12-well plastic dishes and were treated with miRNA mimics, inhibitors or Scrambled. Then, 24 hours after transfection, linear scratch wounds (in triplicate) were created on the confluent cell monolayers using a 200 µL pipette tip. To remove cells from the cell cycle prior to wounding, cells were maintained in serum-free media. To visualize migrated cells and wound healing, images were taken at 0, 24 and 48 h. A total of ten areas were selected randomly from each well, and the cells in three wells from each group were quantified.

For these invasion assays, 24 hours after transfection, 1×10^5^ cells in serum-free media were seeded in transwell migration chambers (8 µm pore size; Millipore, Zürich, Switzerland). The upper chamber of thesetranswell inserts was coated with Matrigel (Sigma-Aldrich, St. Louis, MO, USA). Medium containing 20% FBS was added to the lower chamber. After 24 hours, the non-invading cells were removed with cotton wool. Invasive cells located on the lower surface of the chamber were stained with May-Grunwald-Giemsa stain (Sigma-Aldrich, St. Louis, MO, USA) and then were counted using a microscope (Olympus, Tokyo, Japan).

### Dual luciferase assays

The 3′ UTRs of WASF3 containing these predicted binding sites of miR-217 were amplified using PCR from human cDNA using primers, and inserted into the pMIR-REPORT luciferase reporter vectors (Ambion, Austin, TX, USA) to get the constructs containing the wild-type WASF3 3′UTR (WASF3-WT). WASF3-MUT contained the sequences with mutations in the first putative binding site of WASF3 3′UTR. Mutations of these predicted seed regions in these mRNA sequences were created using the primers including the mutated sequences. The recombination constructs, pRL-TK (Promega, WI, USA) and miR-217 or control mimic were co-transfected into 293T cells using lipofectamine 2000 (Invitrogen, Carlsbad, CA, USA). The plasmid of pRL-TK containing Renilla luciferase was used as the internal control. Firefly and Renilla luciferase activity were measured using Dual Luciferase Assay (Promega) according to the manufacturer's instructions at 24 h after transfection.

### Western blotting analysis

Western blot was performed using standard methods. Total protein was isolated from tumor samples and corresponding normal tissues or cells. The concentration was measured by BCA protein assay kit (Pierce, USA). Proteins were separated by 10% SDS-PAGE, and then transferred to PVDF membranes (Amersham, Buckinghamshire, UK). Membranes were blocked with 5% non-fat dried milk and incubated overnight with anti-WASF3 antibody (Abcam, England); anti-GAPDH antibody (Proteintech, Chicago, USA). After washing with TBST three times, the membranes were incubated for 2 h with goat anti-rabbit antibody (zsgb-bio, Beijing, China).

### Rescue assays of WASF3 gene expression

The full length WASF3 cDNAs (which included theORF and 3′UTR) was PCR-amplified and cloned into the pcDNA3.1 vectorto generate the pcDNA-WASF3 constructs that were used in the rescue assays. The MG-63 cells in 6-well plateswere first transfected with either miR-217 or a scrambled dsRNAs (60 nM). After 24 h in culture, these cells were then co-transfected with miR-217(20 nM) and 2.0 µg pcDNA-WASF3, miR-217 (20 nM) and 2.0 µg pcDNA-empty. Cells were harvested at the indicated time points after hemin addition and were assayed as required.

### Statistical analysis

Each experiment was repeated at least three times. Statistical analyses were performed using SPSS 15.0. Data are presented as the mean ± standard deviation. Statistical analyses were performedwith either an analysis of variance (ANOVA) or Student's t-test and the statistical significance level was set at α = 0.05 (two-side)

## Result

### MiR-217 expression was down-regulated in both osteosarcoma tissues and cell lines

To evaluate the expression of miR-217 in osteosarcoma, qRT-PCR was performed. The expression levels of miR-217 were much lower in tumor cell lines than in hFOB (Figure1A). The expression of miR-217 was also down-regulated in tumor tissues compared to that in non-tumor tissues (Figure 1B and C). The expression of miR-217 in metastaticosteosarcoma tissues were significantly lower than that in non-metastatic tissues. (Figure 1D, p<0.01, independent-samples t test).

**Figure 1:** miR-217 is downregulated in human osteosarcoma cell lines and tissues. (A) Relative expression of miR-217 in four human osteosarcoma cell lines (MG-63, U2OS, SOSP-9607, and SAOS-2) and one normal bone cell line (hFOB) was determined by qRT-PCR. Quantification of miR-217 was measured by qRT-PCR with specific primers for miR-217 and snRNA U6. (B) Relative expression of miR-217 in 60 primary osteosarcoma tissues compared with their pair-matched nontumor tissues. Data areshown as log10 of relative ratio change of osteosarcoma tissues relative tonormal tissues. (C) Relative miR-217expressionlevels in osteosarcoma tissues and adjacent normal regions; (D)The expression of miR-217 in the osteosarcoma tissues from the patients with metastases was lower than that in non-metastases tissues. All data uses t test and is shown as mean ±SEM.

### MiR-217 inhibited osteosarcoma cell proliferation, migration and invasion

To explore the role of miR-217 indevelopment ofosteosarcoma, MG-63 cells were transfected with miR-217 mimics or inhibit with high transfection efficiency (Fig. 2A). The enforced expression of miR-217 led to a significant decrease in the proliferation of the MG-63 cells (Figure 2B). In contrast, the miR-217 inhibitor significantly increased the cell proliferation of the MG-63 cells. The cells treated with miR-217 mimics were distinctively less migratory in comparison tothe scrambled control or untreated cells at 24, and 48 hours after scratching (Fig 2C). Meanwhile, the miR-217 inhibitor significantly accelerated the cell migration of the MG-63 cells. The invasiveness of cells transfected with the miR-217 mimics was significantly decreased compared to the scramble control or untreated cells. And the miR-217 inhibitor significantly increased the cell invasion of the MG-63 cells. (Fig.2D)

**Figure 2:** Overexpression of miR-217 inhibits the osteosarcoma cell line MG-63 proliferation, migration, and invasion. (A) Expression levels of miR-217 were examined by qRT-PCR after transfection of 20 nmol/L of miR-217 mimics, inhibitors or sramble or no transfection in the cell line MG-63. (B) The cells treated with miR-217 mimics, inhibitors or sramble or no transfection were measured by CCK8 assay at different time periods. (C) Wound healing assays of MG-63cells after treatment with miRNA mimics, inhibitors or scramble or no transfection; the relative ratio of wound closure per field is shown. (D) Transwell analysis of MG-63 cells after treatment withmiRNA mimics, inhibitors or scramble or no transfection; the invasive cells per field is shown below, All data uses t test and is shown as mean ±SEM. *p<0.05,** p<0.01, and ***p<0.001.

### WASF3 was the direct target of miR-217 in osteosarcoma

Next, we searched for candidate target genes of miR-217 using publicly available databases; WASF3 was selected for further experimental validation, because the complementary sequence of miR-217 was identified in the 3′UTR of WASF3 mRNA by TargetScan analysis (Fig. 3A). The effect of miR-217 on the translation of WASF3 mRNA into protein was assessed by luciferase reporter assay (Fig. 3B). Overexpression ofmiR-217 remarkably reduced luciferase activity of reporter gene with wild-type, but not mutant WASF3 3′UTR, indicating that miR-217 directly targeted WASF3 3′UTR. Moreover, overexpression of miR-217 reduced the protein but not the mRNA levels of WASF3 in osteosarcoma cells. (Fig. 3C and D).

**Figure 3:** MiR-217 targets WASF3 in osteosarcoma cells. (A) The sequences of miR-217 binding sites within the human WASF3 3′UTR and schematic reporter constructs, in this panel, WASF3-WT represent the reporter constructs containing the entire 3′UTR sequences of WASF3. WASF3-MUT represent the reporter constructs containing mutated nucleotides. (B) The analysis of the relative luciferase activities of WASF3-WT, WASF3-MUT in 293T cells. The error bars are derived from triplicate expriments. (C) qRT-PCR analysis of WASF3 mRNA expression in MG-63 cells after treatment with miRNA mimics or scramble or no transfection. The expression of WASF3 was normalized to GAPDH. (D) Western blot analysis of WASF3 expression in MG-63 cells transfected with miR-217 mimics or scramble or no transfection. GAPDH was also detected as a loading control. All data uses t test and is shown as mean ±SEM.

### Overexpression of WASF3 impaired the miR-217-induced inhibition of proliferation and invasion in osteosarcoma cells

We used rescue experiments to further validate that WASF3 targeting is involved in miR-217-indued anti-tumor properties in osteosarcoma cells. WASF3 expression vectors, pcDNA3.0-WASF3 was used to restore the WASF3 expression. The protein and mRNA level of WASF3 was reduced when miR-217 mimics were transfected with pcDNA-WASF3 after 24 h (Fig. 4A and 4B). As expected, the ectopic expression of WASF3 resulted in a marked increase in cell proliferation, invasion and migration. (Fig. 4C, D, F and G). Inhibition in cell proliferation, invasion and migration by overexpression of miR-217 was significantly attenuated by re-introduction of WASF3 (Fig. 4C, D, F and G). To assess the regulation of miR-217 in the WASF3 expression, the protein level of WASF3 was analyzed in eight miR-217 down-regulated tissues. WASF3 was up-regulated in 8 osteosarcoma tissues compared to their pair-matched adjacent non-tumor tissues. (Fig. 4F)

**Figure 4:** Restore WASF3 expression impairs miR-217-induced inhibition of proliferation and invasion in osteosarcoma cells. (A) Western blot analysis of WASF3 in MG-63 cells co-transfectedwith either miR-217 mimic or scramble and 2.0 µg pCDNA-WASF3 orpCDNA empty vector. (B) The relative WASF3 protein was showed with different combinations. The signal in each lane was quantified using ImageJ software and the ratio of WASF3 to GAPDH was determined. (C) Cell growth curves in MG-63 cells transfected with different combinations using CCK-8 analysis. (D) The relative ratio of wound closure per field with different combinations is shown. (E) Transwell analysis of MG-63 cells treated with different combinations. The invasive cells per field is shown right. (F) Wound healing assays of MG-63 cells after treatment with different combinations. (G) Western blot analysis of WASF3 expression in 8 miR-217 down-regulated osteosarcoma tissues and their pair-matched nontumor tissues. GAPDH was also detected as a loading control. All data uses t test and is shown as mean ±SEM. *p<0.05,** p<0.01,***p<0.001.

## Discussion

Osteosarcoma showed complex genomic changes with a few recurrent chromosomal aberrations, which makes it difficult to identify the molecular features [19]. Recently, accumulating evidences have demonstratedthe role of miRNAs in tumorigenesis and tumor progression of osteosarcoma [20]. miRNAs and their targets genes have been proved to represent potential novel therapeutic biomarkers for osteosarcoma [3], [21], [22]. In this study, we analyzed the expression of miR-217 in 60 osteosarcoma patients and found that miRNAs were much lower in osteosarcoma tissues in comparison with paired adjacent non-tumor bone tissues. Furthermore, we showed that the overexpression of miR-217 in the MG-63 cells reduced cell proliferation. On the other hand, metastasis is the major cause of morbidity and mortality in patients of osteosarcoma; therefore, we investigated the effects of miR-217 on cell migration and invasion. Our result showed that the introduction of miR-217 inhibited the MG-63 cells migration and suppressed cell invasion, further confirming their association with the degree of osteosarcoma malignancy. Moreover, we identified WASF3 as a direct target of miR-217. Our findings, together with those from other groups, suggested that miR-217 played a suppressor role in osteosarcoma tumorigenesis and cell invasion.

In recent years, several miRNAs, such as miR-199b-5b, miR-195, miR-221, miR-183, had been identifiedto be involved in osteosarcoma [23]–[28]. In addition, miR-217 was found to be significantly down-regulated in 21 PDAC patient tissue samples and 7 PDAC cell lines [15]. In agreement with the previous results, we found that miR-217 was down-regulated in 56 cases (56/60, 93%) osteosarcoma tissues compared to in the adjacent tissues.

In this study, we found that restoration of miR-217 significantly inhibited cell proliferation, migration and invasion; and reduced cell viability in osteosarcoma cell lines, indicating that repression of miR-217 might promote tumor progression in osteosarcoma carcinogenesis. Moreover, down-regulation of miR-217 significantly promoted cell proliferation, migration and invasion; enhanced cell viability in osteosarcoma cell lines, indicating that inhibition of miR-217 might promote tumor progression in osteosarcoma carcinogenesis. In conclusion, our results suggested that miR-217 acted as a tumor-suppressor whose downregulation may contribute to the progression of osteosarcoma.

Identification of cancer-specific miRNAs and their targets is pivotal for understanding their roles in tumorigenesis [29], [30]. TargetScan was employed to identify these direct targets of miR-217. WASF3 was predicted as one of the targets of miR-217. Furthermore, overexpression of miR-217 led to a significantly reduction in WASF3 protein and mRNA level and overexpression of miR-217 suppressed WASF3 3′UTR luciferase report activity and this effect was abolished by mutation of the miR-217 seed binding sites. The function of WASF3 was further supported by the observations that inhibition in cell proliferation, invasion and proliferation by overexpression of miR-217 was significantly attenuated by re-introduction of WASF3. These results indicated that miR-217 might function as a tumor suppressor partly by repressing WASF3 expression in osteosarcoma.

The WASF3 gene was a member of the Wiskott Aldrich syndrome family of proteins (WASP), which contained verprolin-cofilin-acidic domains at their C-terminal ends [31], [32]. These domains were thought to coordinate the recruitment of monomeric actin and the ARP2/3 complex of proteins to facilitate actin polymerization, which was essential for cell movement and invasion [32], [33]. Previous studies had shown that inactivation of the WASF3 gene in prostate cancer cells led to suppression of tumorigenicity and metastases [33]. Moreover, activation of WASF3 was required for invasion and lamellipodia formation in breast cancer cells, which was achieved to some extent through its phosphorylation by ABL kinase [34]. WASF3 was previously shown to be required for invasion and metastasis in different cancer cell types and knowckdown of WASF3 led to suppression of invasion and metastasis [35]. In our study, we confirmed that WASF3 was up-regulated in osteosarcoma tissues and overexpression of WASF3 induced osteosarcoma cells proliferation and invasion. However, the relevant mechanisms were still unclear. The ability of miR-217 to target WASF3 might provide one possible mechanism of post-transcriptional control of WASF3.

In conclusion, the current study provided a novel evidence that miR-217 function as a tumor suppressor miRNA in osteosarcoma through repressing WASF3 expression. Based on the association between deregulated miRNA expression and cancers, miRNA-based therapeutic strategies were developed either by restoring the expression or reducing miRNA expression in cancer or, conversely, abrogating overexpressed miRNA. Consequently, our findings provided a molecular basis for the role of miR-217/WASF3 in the progression of human osteosarcoma and suggested that this miRNA could be a potential target for the treatment of osteosarcoma in future.

## Supporting Information

Table S1 **Clinic pathologic charateristics of patients with osteosarcoma.**
(DOC)

Table S2 **Primer sequence.**
(DOC)
